# STAT3 Promotes Invasion and Aerobic Glycolysis of Human Oral Squamous Cell Carcinoma via Inhibiting FoxO1

**DOI:** 10.3389/fonc.2019.01175

**Published:** 2019-11-05

**Authors:** Min Zheng, Ming-xin Cao, Xiang-hua Yu, Li Li, Ke Wang, Sha-sha Wang, Hao-fan Wang, Ya-Jie Tang, Ya-ling Tang, Xin-hua Liang

**Affiliations:** ^1^Department of Stomatology, Zhoushan Hospital, Wenzhou Medical University, Zhoushan, China; ^2^State Key Laboratory of Oral Diseases and National Clinical Research Center for Oral Diseases, Department of Oral and Maxillofacial Surgery, West China Hospital of Stomatology, Sichuan University, Chengdu, China; ^3^State Key Laboratory of Microbial Technology, Shandong University, Qingdao, China; ^4^State Key Laboratory of Oral Diseases and National Clinical Research Center for Oral Diseases, Department of Oral Pathology, West China Hospital of Stomatology, Sichuan University, Chengdu, China

**Keywords:** STAT3, FoxO1, aerobic glycolysis, EMT, OSCC

## Abstract

Signal transducer and activator of transcription 3 (STAT3), a previously accepted tumor-promoting protein in various malignancies, plays a key role in the process of cancer glycolysis. However, the role and potential mechanism of STAT3 in aerobic glycolysis and progression of oral squamous cell carcinoma (OSCC) has not been explored. In the present study, we demonstrated that STAT3 knockdown remarkably inhibited migration, invasion, expressions of epithelial-mesenchymal transition (EMT) markers, and aerobic glycolysis of OSCC cells by up-regulation of FoxO1. Consistently, the expression of nuclear Tyr705-phosphorylated STAT3, an active form of STAT3, was significantly elevated in OSCC tissues compared with adjacent normal tissues, and increased nuclear staining of Tyr705-phosphorylated STAT3 was associated with metastasis and shorter overall survival. Moreover, FoxO1, which was also mainly expressed in OSCC specimens, decreased in poorly-differentiated tissues compared with the relatively well-differentiated ones, and inversely correlated with the expression of nuclear Tyr705-phosphorylated STAT3 from patients with OSCC. Hence, our findings collectively characterized the contributing role of STAT3/FoxO1 in invasion and aerobic glycolysis of OSCC cells, which may lead to the worse clinical outcome.

## Introduction

Oral squamous cell carcinoma (OSCC), which includes epithelial malignancies of the oral cavity and oropharynx, is one of the most prevalent problems in many parts of the world (1, 2). Despite improvements in diagnosis and therapeutics in recent years, the mortality rate of OSCC is still high mainly due to the lack of early detection markers, recurrence and metastases, which account for ~90% of all cancer deaths (3, 4). Thus, it is essential to thoroughly identify the biomarkers and therapeutic targets of OSCC for future clinical applications.

Metastasis, a dynamic process which is multifactorial and involves the detachment of cancer cells from the primary site, cell mobility, entry of lymphatic and vascular vessels, and recolonization conceptually, is a major cause of poor prognosis (5, 6). During this process, epithelial-mesenchymal transition (EMT) is considered as a critical mechanism for cancer cells to become invasive. It is well-established that during EMT, epithelial cells transit to mesenchymal phenotype that leads to the enhanced cell migration, invasion, and initiation of metastasis (7, 8). Accumulating evidence suggests that these cells reprogram metabolism with higher aerobic glycolysis to meet the elevated bioenergetic and biosynthetic requirements for growth and metastasis of cancer (9, 10).

Signal transducer and activator of transcription 3 (STAT3) is a member of the STAT protein family, and is known for its roles in promoting tumor cells proliferation, survival, tumor invasion, angiogenesis, and immunosuppression (11, 12). Activated by members of the IL-6 family cytokines, receptor tyrosine kinases, activated JAKs, or oncogenic cellular tyrosine kinases, STAT3 proteins are continuously phosphorylated in tumors, mainly at Y705, and translocate to the nucleus to exert tumor-promoting effects primarily acting as transcription factors (13). Recently, STAT3 was also found to have important roles in tumor glycolysis. In a study of head and neck squamous cell carcinoma, decreased STAT3 expression was accompanied with increased oxygen consumption, and reduced aerobic glycolysis owing to GRIM-19 overexpression, while the specific mechanism of STAT3 resulting in abnormal glycolysis was unclear (14). Another study reported that STAT3 could promote aerobic glycolysis of hepatocellular carcinoma cells via targeting and increasing hexokinase 2 (15). However, STAT3 signaling pathway was investigated to suppress aerobic glycolysis of breast cancer cells HeLa and MCF-7, thus promoting their apoptosis mediated by PSA (16).

In the present study, we characterized the function of STAT3 in OSCC cells, and carried out immunohistochemical analysis of pY-STAT3 protein (at the 705 residue) in OSCC tissues to determine its relationships with clinicopathological features and prognosis. The data revealed that STAT3 promoted migration, invasion, EMT and aerobic glycolysis of OSCC cells by inhibiting FoxO1 transcription. Then, we found that Tyr705-phosphorylated STAT3 was correlated with metastasis and poor prognosis of OSCC patients, and inversely correlated with FoxO1 expression, demonstrating the clinical significance of STAT3/FoxO1 during OSCC progression.

## Materials and Methods

### Patients and Clinical Specimens

The present study was approved by the Institutional Ethics Committee of the West China Medical Center, Sichuan University, China. Sixty eight patients diagnosed with OSCC in West China School of Stomatology, Sichuan University between 2000 and 2003 were recruited after giving informed consent. Primary resection and no prior treatment had been giving to patients in the present study. Besides, 10 cases of normal oral mucosae were included in this study. All specimens were fixed in 10% formaldehyde, then embedded in paraffin, and confirmed by hematoxylin-eosin staining.

### Reagents

Monoclonal mouse anti-human antibodies to STAT3 (sc-293151), FoxO1 (H-128), β-catenin (sc-1496) were purchased from Santa Cruz Biotechnology Inc. (Santa Cruz, CA, USA). Monoclonal mouse anti-human antibodies to tyrosine phosphorylated STAT3 (pY-STAT3, at the 705 residue) (9145S), E-cadherin (3195S) were obtained from Cell Signaling Technology Inc. (Danvers, MA, USA). Monoclonal mouse anti-human antibodies to N-cadherin (ab98952), Vimentin (ab8978) were purchased from Abcam (Cambridge, MA, USA). Monoclonal mouse anti-human antibody to β-actin (ab008-100) was purchased from MultiSciences (Hangzhou, China).

### Immunohistochemistry

All sections were deparaffinized in xylene and rehydrated through a gradient alcohol series. After endogenous peroxidase activity blocking by incubation with 3% hydrogen peroxide for 20 min, antigen retrieval by 0.01 M citrate buffer (pH = 6.0) in a microwave oven for 3 min, and non-specific binding blocking by incubation with 5% normal goat serum for 25 min, sections were incubated with primary pY-STAT3 antibody (1:100) at 4°C overnight in a moist chamber. The sections were then incubated with biotinylated anti-mouse IgG and streptavidin-biotin peroxidase. The primary antibody was detected using diaminobenzidine tetrahydrochloride (DAB), and sections were counterstained with hematoxylin. Six microscopic fields at 200× magnification per section were observed and at least 1,000 cells were counted independently by three of us. The percentage of cells showing positive staining was classified into lower and higher part due to the median for all cases. For representing negative expression, weakly positive expression, moderately positive expression and strongly positive expression, the percentage was categorized into (–), <5%; (+), 5–25%; (++), 25–50%; (+ + +), >50%. In negative controls, the primary antibody was replaced with isotype-specific immunoglobulin (IgG) to ensure specificity.

### Cell Lines and Transfections

In present study, human OSCC cell lines Cal-27, Tca8113, and SCC25 were obtained from State Key Laboratory of Oral Diseases, Sichuan University. Cells were cultured in Dulbecco's modified Eagle's medium (DMEM; Hyclone, Logan, UT, USA) containing 10% FBS in a humidified atmosphere of 95% air and 5% CO2 at 37°C. For transfections, targeted sequences of shRNAs were as follows: STAT3: GCACAATCTACGAAGAATCAA (sh-1-S), GGTTGCTGGTCAAATTCCCTGAGTT (sh-2-S), and AAGGAGGAGGCATTCGGAAAGTATT (sh-3-S); FoxO1: GCATGTTCATTGAGCGCTTAG (sh-1-F), CAATTCGTCATAATCTGTCCCTACA (sh-2-F), and CAACCTTCTCTCATCACCAACATCA (sh-3-F); scramble: TTCTCCGAACGTGTCACGTAA. The shRNA lentiviral vector pHBLV-U6-mCherry-Puro and the human STAT3 gene stably overexpressing vector using vector pDC316-mCMV-mCherry-Puro was from Hibio (Hangzhou, China), and all constructs were verified by sequencing. Cells were transfected with shRNAs in the presence of 5 μg/ml of polybrenen and incubated for 12 h. Then, 2 μg/ml puromycin was used to select transfected cells for 7 days. Transfected cells were collected and verified by qRT-PCR and Western blot, and thus for further experiments.

### qRT-PCR

Total RNA was extracted using Trizol reagent (Invitrogen, Carlsbad, CA, USA). The reverse transcription was performed with HiScript II Q RT SuperMix for qPCR (Vazyme, Nanjing, China). The real-time PCR reaction was carried out with ChamQ™ SYBR Color qPCR Master Mix (Vazyme) on CFX Connect Real-Time System (Bio-Rad, Hercules, CA, USA) according to the protocol. Specific primers were listed in Supplementary Data. And the relative expression of target genes was represented using 2^−ΔΔCT^ method.

### Western Blot

The whole cells extracts were lysed using 200 μl RIPA lysis buffer (Santa Cruz) for 30 min. Equal amounts of protein were then separated on SDS-PAGE, transferred to PVDF membranes (Millipore, Billerica, MA, USA), and immunoblotted with primary antibody. Antibodies against STAT3, pY-STAT3, FoxO1, E-cadherin, N-cadherin, β-catenin, Vimentin, and β-actin were used at a 1:1,000 dilution. Immunoblots were visualized after using goat anti-mouse antibody (MultiSciences) with the chemiluminescence (ECL) reagent (Beyotime Biotechnology, Shanghai, China) and ChemiDoc XRS+ System (Bio-Rad).

### Wound Healing Assay

Cells were seeded in a 6-well plate until forming confluent monolayers. Twelve hours prior to the experiment, cells were starved in serum-free DMEM medium. All cells were then scratched with a pipette tip to form a gap space. Finally, photomicrographs were taken immediately after the scratch, and after 24 h. The closed scratch areas were measured using ImageJ software. Each assay was carried out in triplicate.

### Cell Invasion Assay

Cell invasion assay was performed using 24-well plates (pore size 8 μm; Millipore). Cells were starved in serum-free DMEM medium for 12 h. Then 5.0 × 10^4^ cells were seeded in the upper chamber coated with Matrigel (BD Bioscience, San Diego, CA, USA). Complete medium was added to the lower chamber. After 24 h incubation and 0.1% crystal violet staining, cells that had invaded through the Matrigel were counted under a microscope in five pre-determined fields (×200). Experiments were carried out in triplicate.

### Flow Cytometry-Based Apoptosis Analysis

Cell apoptosis was measured using the Annexin V-FITC Apoptosis Detection Kit (Invitrogen). Cells were grown in 6-well plates and resuspended in 1× Binding Buffer after 48 h. Five microliter of Annexin FITC Conjugate and 10 μl of Propidium Iodide Solution were added into each cell suspension, separately. Then, we analyzed the stained cells using a flow cytometry (FACScalibur, Becton-Dickinson).

### Glucose Consumption and Lactate Production Assays

The glucose consumption and lactate production levels were detected using Glucose (Rongsheng Biotechnology, Shanghai, China) and Lactate (Abcam) assay kits according to the protocol. Results were normalized to 10^5^ cells.

### Statistical Analysis

Chi-square was used to analyze associations between related factors. Kaplan-Meier method was used to estimate survival curves, and differences between two groups were evaluated using log-rank test. The correlation between pY-STAT3 and FoxO1 expression in OSCC specimens was assessed by 2-tailed Pearson's statistics. Means comparisons were analyzed using Student *t*-test or one-way ANOVA. Experimental values were expressed as means ± SD. *P* < 0.05 was considered to be statistically significant.

## Results

### STAT3 Knockdown Inhibits Migration, Invasion Potential, and EMT of OSCC Cells

To investigate the role of STAT3 in migration, invasion and EMT of OSCC cells, we firstly assessed the relative STAT3 mRNA expression in five OSCC cell lines, including SCC25, Cal-27, HSC3, Tca8113, and UM1 (Figure 1A). Cal-27 and Tca8113 were selected for further experiments due to their higher STAT3 expressions. Then, we applied short hairpin RNAs (shRNAs) to knockdown STAT3 expression in Cal-27 and Tca8113 cells and selected sh-2-STAT3 which had the highest knockdown efficiency for further experiments (Supplementary Figure 1). As confirmed by Western blot and qRT-PCR, the expression of STAT3 was decreased significantly (Figure 1B). Using wound healing assay, down-expression of STAT3 remarkably decreased the wound closure of Cal-27 cells and Tca8113 cells (Figure 1C). And according to cell invasion assay, invasive abilities of Cal-27 and Tca8113 cells were greatly decreased after inhibiting STAT3 expression (Figure 1D). Upregulation of STAT3 in SCC25 cells confirmed its roles in facilitating invasiveness using wound healing and cell invasion assays (Supplementary Figure 2).

**Figure 1:** STAT3 knockdown inhibits migration, invasion potential, and EMT in OSCC cells. **(A)** STAT3 mRNA levels were evaluated using qRT-PCR in SCC25, Cal-27, HSC3, Tca8113, and UM1 cells. **(B)** STAT3 expression was detected by qRT-PCR and Western blot after transfected with STAT3 shRNA in OSCC cells. **(C)** Images of the wound closure of monolayer Cal-27 and Tca8113 cells with STAT3 knockdown at the time point of 0 and 24 h are presented on the left. Quantitative results are illustrated on the right. **(D)** The effect of STAT3 knockdown on OSCC cells invasion were determined by Transwell assay with Matrigel, and the representative images are on the left. Quantitative results are illustrated on the right. **(E)** The effects of Cal-27-STAT3 knockdown on expressions of EMT markers, E-cadherin, N-cadherin, β-catenin, and Vimentin, were measured using qRT-PCR and Western blot. β-actin was used as a loading control. **(F)** Flow cytometry was used to examine the percentage of apoptotic cells in Cal-27 cells with STAT3 knockdown and scramble control cells. All assays were carried out in triplicate. Results were shown as means ± SD. *P < 0.05.

As EMT is a key process for cancer cell migration and invasion, defined by loss of epithelial cell polarity and reorganization of the cytoskeleton, and STAT3 is activated in tumors as the form of pY-STAT3 (17), we next examined the expression of epithelial and mesenchymal markers of EMT and pY-STAT3 protein expression in STAT3-inhibited Cal-27 cells. We found that STAT3 knockdown significantly decreased expression of pY-STAT3, and knockdown of STAT3 led to increased expressions of E-cadherin and β-catenin, and suppressed expressions of N-cadherin and Vimentin both in protein and in mRNA levels by Western blot and qRT-PCR (Figure 1E). However, no obvious changes were found in cell apoptosis after STAT3 down-regulation by flow cytometry (Figure 1F). This indicated that down-expression of STAT3 significantly inhibited migration, invasion and EMT of OSCC cells, with no effect on cell apoptosis.

### STAT3 Knockdown Inhibits Aerobic Glycolysis of OSCC Cells

Aerobic glycolysis, widely recognized as a central hallmark of human cancer, facilitates survival of aggressive cancer cells as well as their metastasis through metabolic pattern shifting (18). Using Glucose consumption and Lactate production assays, we found that down-expression of STAT3 led to remarkably decreased glucose consumption and lactate production, both in Cal-27 and in Tca8113 cells (Figures 2A,B). Moreover, qRT-PCR analysis showed that knockdown of STAT3 attenuated the mRNA expression of glycolysis-related genes, including PKM2 and LDHA, in Cal-27 and Tca8113 cells (Figures 2C,D). Thus, we speculated that STAT3 promoted aerobic glycolysis of OSCC cells, which might provide a competitive environment for OSCC cells migration and invasion.

**Figure 2:** STAT3 knockdown inhibits aerobic glycolysis in OSCC cells. **(A)** Glucose consumption assay was used to detect the glucose consumption in STAT3-knockdown Cal-27 and Tca8113 cells. The data showed that down-regulation of STAT3 led to lower glucose consumption in Cal-27 and Tca8113 cells. **(B)** Lactate production assay was used to detect the lactate production in STAT3-knockdown Cal-27 and Tca8113 cells. The data showed that down-regulation of STAT3 led to lower lactate production in Cal-27 and Tca8113 cells. **(C)** PKM2 mRNA levels in STAT3-knockdown Cal-27 and Tca8113 cells were examined by qRT-PCR. **(D)** LDHA mRNA levels in STAT3-knockdown Cal-27 and Tca8113 cells were examined by qRT-PCR. Each assay was carried out in triplicate. Results were shown as means ± SD. *P < 0.05.

### Transcription of FoxO1 Was Regulated by STAT3 in OSCC Cells

As a downstream protein of STAT3 signaling pathway, FoxO1 has been demonstrated to play important biological roles as tumor suppressor in regulating cancer cell growth, apoptosis, DNA damage repair, and so on (19, 20). Emerging researches have also showed that FoxO1 is a critical glucose metabolism-related protein (21). Thus, we evaluated whether FoxO1 was regulated by STAT3 in OSCC cells. As shown in Figures 3A,B, FoxO1 expression was elevated in STAT3 knockdown Cal-27 and Tca8113 cells, both in protein and in mRNA levels, indicating that STAT3 inhibited FoxO1 transcription in OSCC cells.

**Figure 3:** The transcription of FoxO1 was inhibited by STAT3 in OSCC cells. **(A)** FoxO1 protein levels in STAT3-knockdown Cal-27 and Tca8113 cells were examined by Western blot. **(B)** FoxO1 mRNA levels in STAT3-knockdown Cal-27 and Tca8113 cells were examined by qRT-PCR. Results were shown as means ± SD. *P < 0.05.

### FoxO1 Knockdown Promotes Migration, Invasion Potential, and EMT of OSCC Cells

To further evaluate the role of FoxO1, we applied shRNAs to knockdown FoxO1 expression in Cal-27 and Tca8113 cells, and using Western blot and qRT-PCR, we selected sh-1-FoxO1 which had the highest knockdown efficiency for further experiments (Supplementary Figure 1; Figure 4A). As shown in Figures 4B,C, wound healing and cell invasion assay revealed that down-expression of FoxO1 significantly promoted the wound closure and invasive abilities of OSCC cells. Then we examined the EMT markers after FoxO1 knockdown using Western blot and qRT-PCR in Cal-27 cells. Results showed that the expressions of E-cadherin and β-catenin were decreased, while the expressions of N-cadherin and Vimentin were increased, both in mRNA and in protein levels. Moreover, after co-transfecting Cal-27 cells with sh-2-STAT3 and sh-1-FoxO1, mRNA levels of E-cadherin and β-catenin were decreased, N-cadherin and Vimentin were increased compared to those in sh-2-STAT3 and scramble co-transfected cells, which provided more evidence that FoxO1 knockdown could reverse the anti-invasive effects caused by STAT3 down-regulation (Figure 4D). However, no evident changes were found in cell apoptosis after FoxO1 knockdown (Figure 4E). These indicated that FoxO1 could inhibit migratory and invasive ability of OSCC cells as downstream protein of STAT3.

**Figure 4:** FoxO1 knockdown promotes migration, invasion potential, and EMT in OSCC cells. **(A)** FoxO1 expression was detected by qRT-PCR and Western blot after transfected with FoxO1 shRNA in OSCC cells. **(B)** Images of the wound closure of monolayer Cal-27 and Tca8113 cells with FoxO1 knockdown at the time point of 0 and 24 h are presented on the left. Quantitative results are illustrated on the right. **(C)** The effect of FoxO1 knockdown on OSCC cells invasion were determined by Transwell assay with Matrigel, and the representative images are on the left. Quantitative results are illustrated on the right. **(D)** The effects of Cal-27-FoxO1 knockdown on expressions of EMT markers, E-cadherin, N-cadherin, β-catenin, and Vimentin, were measured using qRT-PCR and Western blot. And the effects of Cal-27-sh-2-STAT3/sh-1-FoxO1 on expressions of EMT markers, E-cadherin, N-cadherin, β-catenin, and Vimentin, were measured using qRT-PCR compared with those of sh-2-STAT3/scramble group. β-actin was used as a loading control. **(E)** Flow cytometry was used to examine the percentage of apoptotic cells in Cal-27 cells with FoxO1 knockdown and scramble control cells. All assays were carried out in triplicate. Results were shown as means ± SD. *P < 0.05.

### FoxO1 Knockdown Facilitates Aerobic Glycolysis of OSCC Cells

Then we investigated the effect of FoxO1 knockdown on aerobic glycolysis of OSCC cells. As shown in Figures 5A,B, using Glucose consumption and Lactate production assays, down-expression of FoxO1 led to increased glucose consumption and lactate production in Cal-27 and Tca8113 cells, reversing the effects of sh-2-STAT3 in inhibiting glucose consumption and lactate production. The mRNA expressions of glycolysis-related genes, PKM2 and LDHA, were also up-regulated in FoxO1-knockdown, or FoxO1 and STAT3 co-knockdown Cal-27 and Tca8113 cells, compared to those in scramble, or sh-2-STAT3/scramble transfected cells, respectively (Figures 5C,D). Therefore, these data suggested that STAT3 contributed to invasion and aerobic glycolysis of OSCC cells mediated by down-regulation of FoxO1.

**Figure 5:** FoxO1 knockdown promotes aerobic glycolysis in OSCC cells. **(A)** Glucose consumption assay was used to detect the glucose consumption in Cal-27 and Tca8113 cells transfected with scramble, sh-1-FoxO1, sh-2-STAT3/scramble, or sh-2-STAT3/sh-1-FoxO1. The data showed that down-regulation of FoxO1, or both FoxO1 and STAT3 led to higher glucose consumption in Cal-27 and Tca8113 cells. **(B)** Lactate production assay was used to detect the lactate production in Cal-27 and Tca8113 cells transfected with scramble, sh-1-FoxO1, sh-2-STAT3/scramble, or sh-2-STAT3/sh-1-FoxO1. The data showed that down-regulation of FoxO1, or both FoxO1 and STAT3 led to higher lactate production in Cal-27 and Tca8113 cells. **(C)** PKM2 mRNA levels in Cal-27 and Tca8113 cells transfected with scramble, sh-1-FoxO1, sh-2-STAT3/scramble, or sh-2-STAT3/sh-1-FoxO1 were examined by qRT-PCR. **(D)** LDHA mRNA levels in Cal-27 and Tca8113 cells transfected with scramble, sh-1-FoxO1, sh-2-STAT3/scramble, or sh-2-STAT3/sh-1-FoxO1 were examined by qRT-PCR. Each assay was carried out in triplicate. Results were shown as means ± SD. *P < 0.05.

### Analysis of Tyr705-Phosphorylated STAT3 Expression, Clinical Significance, and Correlation With FoxO1 in OSCC Patients

To address whether STAT3 was associated with FoxO1 in OSCC patients, we first evaluated expressions of Tyr705-phosphorylated STAT3 in OSCC specimens. Using immunohistochemistry analysis, we showed that Tyr705-phosphorylated STAT3 was overexpressed in OSCC compared to normal adjacent tissues (Figure 6A). Nuclear staining for Tyr705-phosphorylated STAT3 was 3.2 ± 1.92 (%) of the normal tissues and 42.18 ± 25.27 (%) of the tumor tissues, respectively. And OSCC patients with negative, weak, moderate, and strong expression of Tyr705-phosphorylated STAT3 were 10.3% (7/68), 20.6% (14/68), 22.1% (15/68), 47.1% (32/68), separately (Figure 6B; Table 1). Then patients were divided into higher and lower Tyr705-phosphorylated STAT3 expression groups with the cutoff point of 48% (nearly the median of percentage for all OSCC cases in our study which was 47.64%) in order to estimate the relationship between Tyr705-phosphorylated STAT3 and overall survival of OSCC patients. Kaplan-Meier survival analysis revealed that patients with a higher Tyr705-phosphorylated STAT3 expression in tumor tissues had a significantly reduced overall survival (*p* = 0.041) (Figure 6C). Furthermore, significant correlations were found between higher Tyr705-phosphorylated STAT3 expression and higher tumor size (*p* = 0.048), poorer differentiation (*p* < 0.000), higher clinical stage (*p* = 0.002), and the presence of lymph node metastasis (*p* = 0.010), while no obvious relations were found between Tyr705-phosphorylated STAT3 and age, gender, drink, smoke, and recurrence in this study (Table 2).

**Figure 6:** Representative micrographs of Tyr705-phosphorylated STAT3 and FoxO1 in OSCC tissues and adjacent normal tissues by immunohistochemistry. **(A)** Images showed few expressions of Tyr705-phosphorylated STAT3 in adjacent normal tissues and high levels of nuclear expressions of Tyr705-phosphorylated STAT3 in OSCC tissues, and few expressions of FoxO1 in adjacent normal tissues, while higher level of nuclear and cytoplasmic staining of FoxO1 in relatively well-differentiated OSCC tissues than in poorly-differentiated tissues. Magnifications: 100× for the left; 200× for the middle; 400× for the right. Scale bar, 50 μm. **(B)** The distribution of OSCC patients with different positive rates of Tyr705-phosphorylated STAT3 and FoxO1 expression. For representing negative expression, weakly positive expression, moderately positive expression, and strongly positive expression in immunohistochemistry results of OSCC specimens, the percentage was categorized into (–), <5%; (+), 5–25%; (++), 25–50%; (+ + +), >50%. **(C)** Patients with a higher Tyr705-phosphorylated STAT3 expression in the tumors (*n* = 33) had a significantly reduced overall survival rate compared to those with a lower level of expression (*n* = 35) (*P* = 0.041). And patients with a higher FoxO1 expression (*n* = 34) in tumor tissues had a significantly increased overall survival rate (*p* = 0.0003). **(D)** 2-tailed Pearson's statistics showed that Tyr705-phosphorylated STAT3 expressions were significantly inversely associated with FoxO1 expressions (*p* < 0.0001, *r* = −0.4637).

**Table 1:** The expression of Tyr705-phosphorylated STAT3 and FoxO1 in normal oral mucosa and OSCC.

	**Tyr705-phosphorylated STAT3**		**FoxO1**	
**Cases**	**Normal** **(*n* = 10)**	**OSCC** **(*n* = 68)**	**Normal** **(*n* = 10)**	**OSCC** **(*n* = 68)**
−	7	7	9	27
+	3	14	1	33
++	0	15	0	6
+++	0	32	0	2
*p* value	<0.000^*^		0.030^*^	

*(−), <5% negative expression; (+), 5–25% weakly positive expression; (++), 25–50% moderately positive expression; (+++), >50% strongly positive expression*.

* *p < 0.05 was regarded as statistically significant in Chi square test*.

**Table 2:** Clinicopathological features of OSCC patients and their relationship with Tyr705-phosphorylated STAT3 expression (*n* = 68).

**Characteristics**	**Cases**	**Tyr705-phosphorylated STAT3**		***p* value**
		**Higher (≥54%)**	**Lower (<54%)**	
**Age (years)**				
<60	31	17	14	0.341
≥60	37	16	21	
**Gender**				
Female	29	14	15	0.572
Male	39	19	20	
**Drink**				
Yes	45	25	20	0.105
No	23	8	15	
**Smoke**				
Yes	42	20	22	0.849
No	26	13	13	
**Tumor size**				
T1–T2	20	6	14	0.048^*^
T3–T4	48	27	21	
**Differentiation**				
Well	30	4	26	<0.000^*^
Moderate	21	14	7	
Poor	17	15	2	
**Clinical stage**				
I–II	18	3	15	0.002^*^
III–IV	50	30	20	
**Nodal metastasis**				
Yes	19	14	5	0.010^*^
No	49	19	30	
**Recurrence**				
Yes	13	8	5	0.297
No	55	25	30	

* *p < 0.05 was regarded as statistically significant in Chi square test*.

Additionally, immunohistochemical staining of FoxO1 was also carried out in OSCC specimens and normal tissues. We found that it was more expressed in OSCC than in normal adjacent tissues. OSCC patients with negative, weak, moderate, and strong expression of FoxO1 were 39.7% (27/68), 48.5% (33/68), 8.8% (6/68), 2.9% (2/68), respectively (Figure 6B; Table 1). FoxO1 expression was observed in both nucleus and cytoplasm, and there was a significant decrease in poorly-differentiated tissues compared with relatively well-differentiated tissues (Figure 6A). Then Kaplan-Meier survival analysis revealed that patients with a higher FoxO1 expression (FoxO1 ≥ 7.5%, *n* = 34) in tumor tissues had a significantly increased overall survival (*p* = 0.0003) (Figure 6C). Furthermore, we assessed the correlation between expression of Tyr705-phosphorylated STAT3 and FoxO1. Remarkably, Tyr705-phosphorylated STAT3 expression was significantly inversely associated with FoxO1 expression (*p* < 0.0001, *r* = −0.4637, Figure 6D). These data suggested that Tyr705-phosphorylated STAT3 might be a potential biomarker for poor prognostic prediction in OSCC patients and inversely correlated with FoxO1. Negative controls with IgG were conducted to prevent the false positives (Supplementary Figure 3).

## Discussion

STAT3 has a contributing role in most human malignancies, where it not only promotes proliferation, survival, angiogenesis, and metastasis, but also interferes with apoptosis and immunosuppression (22, 23). It has also been shown that STAT3 promotes initiation and malignant progression of OSCC (24–26). Yang and colleagues demonstrated that STAT3 promoted proliferation and suppressed apoptosis in OSCC cells. Other reports also revealed that STAT3 participated in the development of OSCC under the regulation of non-coding RNAs let-7a or MALAT1. Consistent with these reports, we observed that knockdown of STAT3 inhibited migratory and invasive abilities of OSCC cells. As EMT, characterized by repression of epithelial markers and production of mesenchymal markers, increased in cell migration and invasion of various epithelial cancers, we then found that STAT3 knockdown in OSCC cells led to increases of E-cadherin and β-catenin, and decreases of N-cadherin and Vimentin, both in mRNA and protein levels. These were in line with a previous study showing that STAT3 promoted migration and invasion of OSCC and altered the expression of EMT markers mediated by EZH2/miR-200 axis both *in vitro* and *in vivo* (27).

STAT3 exerts effects mainly by translocating into the nucleus and interacting with specific DNA binding elements, thus impacting transcription. The process of nuclear accumulation is strongly dependent on Tyr705 phosphorylation, while other reports also showed that STAT3 could enter the nucleus independent of its phosphorylation (28, 29). However, phosphorylated STAT3 proteins shuttle more rapidly than inactivated ones, indicating the fact that STAT3 is continuously activated in most tumors. Although within the STAT3 lies another phosphorylation site, serine 727, whose phosphorylation also demonstrated gene regulation after nuclear translocation, nuclear accumulation and STAT3 activating are strongly dependent on Tyr705, but not Ser727 phosphorylation (12, 13). In addition, a study concerning the immunohistochemical levels of STAT3 (tyrosine/serine) in OSCC specimens have reported that pSTAT3 at Tyr705 showed a significant higher percentage, intensity levels in poorer differentiated tumor, while pSTAT3 at Ser727 did not appear to correlate with tumor differentiation (30). Thus, we examined Tyr705 phosphorylation of STAT3 in this study to show the nuclear transport and transcriptional activity of STAT3. We observed Tyr705-phosphorylated STAT3 overexpression in the OSCC tissues compared to their expression in normal tissues, and this overexpression was correlated with metastasis and poor prognosis of OSCC patients. Hence, these results demonstrated that STAT3 contributed to the progression of OSCC.

Despite a high genetic diversity, cancer cells still exhibit a common set of characteristics, continuous high glucose uptake and a higher rate of aerobic glycolysis than that in normal cells, to meet the rapid energy requirements for activities like EMT and progression (31, 32). In this study, we found that STAT3 promoted aerobic glycolysis of OSCC cells by elevating glucose consumption and lactate production, and contributed to increased migration, invasion, and EMT process. This is in line with previous reports. In a study of head and neck squamous cell carcinoma, elevated expression of GRIM-19 could lead to increased oxygen consumption, and reduced aerobic glycolysis and cell proliferation, accompanying decreased STAT3 expression (14). Additionally, STAT3 could promote aerobic glycolysis of hepatocellular carcinoma cells via targeting and increasing hexokinase 2 (15). However, in another study, STAT3 signaling pathway could suppress aerobic glycolysis of breast cancer cells HeLa and MCF-7, thus promoting their apoptosis mediated by PSA (16). These may due to the different tumor microenvironment and the importance of STAT3 in aerobic glycolysis regulation in OSCC needs to be explored further.

FoxO1, one of the members of the Forkhead box O-class proteins, was considered as a downstream factor of STAT3 (33). In a study of bladder cancer, miR-145 inhibited STAT3 phosphorylation at Tyr705 through targeting JAK2 mRNA coding sequence, a crucial upstream kinase of STAT3, thus enhancing FoxO1 promoter transcription and inhibiting tumor growth (34). And in breast cancer cell lines, combination therapy of trastuzumab and MPA markedly decreased constitutive activation of STAT3 and resulted in higher expression of proapoptotic factors such as p27 and FoxO1 (35). The data were in line with our findings that STAT3 inhibition in OSCC cells led to increased FoxO1 mRNA and protein levels and FoxO1 expression was inversely correlated with p-STAT3 expression in OSCC tissues. However, a previous study has showed that STAT3 could promote T-cell survival and inhibit IL-2 production via binding directly to FoxO1 promoter and up-regulating FoxO1 expression (36). This interaction difference may be due to the distinct types of cells population.

As a tumor-suppressor protein which has pleiotropic functions including inhibiting cell proliferation, inducing apoptosis, protecting cells from oxidative stress and DNA damage, and regulating immune response, FoxO1 is also a critical glucose metabolism-related protein (20, 21, 37, 38). In hepatic FoxO1/3/4 knockout mice, the overall glucose phenotype was altered with decreased gluconeogenesis and increased glycolysis (39). In vascular endothelial cells, FoxO1 decelerated metabolic activity by reducing glycolysis and mitochondrial respiration, mediated by inhibition of MYC, a powerful driver of anabolic metabolism and growth (40). However, the metabolism-related effects of FoxO1 in OSCC microenvironment have not been developed. In this study, we found that FoxO1 was highly expressed in OSCC than in normal tissues, while FoxO1 expression decreased in poor-differentiated OSCC compared with the relatively well-differentiated tissues, which suggests that FoxO1 might be activated during tumorigenesis and could prevent OSCC from becoming more aggressive. Results also showed that FoxO1 inhibition in OSCC cells promoted migration, invasion, and EMT with increased aerobic glycolysis, suggesting that FoxO1 partially participated in the STAT3 regulatory pathway of promoting invasion and aerobic glycolysis of OSCC cells.

In conclusion, we clarified that STAT3 promoted migratory and invasive phenotypes, EMT, and aerobic glycolysis of OSCC cells by inhibiting FoxO1 transcription. Consistently, clinical studies have revealed that Tyr705-phosphorylated STAT3 was up-regulated in cancer tissues and correlated with metastasis and poor prognosis. These findings provided the evidence of STAT3/FoxO1 for the first time in modulating glycolysis to promote the malignant transformation of OSCC. Considering that tumors are generally typified by phenotypic diversity, it would be interesting in the future to unravel the metabolic heterogeneity and flexibility that will contribute to the utility of STAT3/FoxO1-targeted therapy for better OSCC management.

## Data Availability Statement

The datasets used and analyzed during the current study are available from the corresponding author on reasonable request.

## Ethics Statement

The studies involving human participants were reviewed and approved by the Institutional Ethics Committee of the West China Medical Center, Sichuan University, China. The patients/participants provided their written informed consent to participate in this study.

## Author Contributions

MZ, MC, XY, YT, and XL designed the research study. MZ, MC, XY, and LL conducted the cell experiments. MZ, MC, XY, SW, HW, and Y-JT conducted the experiments on the human samples. MZ, MC, YT, and XL were involved in data analysis. MZ and MC were responsible for writing of manuscript. All authors reviewed the manuscript.

### Conflict of Interest

The authors declare that the research was conducted in the absence of any commercial or financial relationships that could be construed as a potential conflict of interest.

## Supplementary Material

Supplementary Figure 1 The knockdown efficiency of shRNAs targeting STAT3 and FoxO1. **(A)** The STAT3 mRNA levels after using three kinds of sh-STAT3s in Cal-27 and Tca8113 cells. **(B)** The FoxO1 mRNA levels after using three kinds of sh-FoxO1s in Cal-27 and Tca8113 cells. Each assay was carried out in triplicate. Results were shown as means ± SD. ^*^*P* < 0.05.

Supplementary Figure 2 STAT3 overexpression promotes migration, and invasion potential in OSCC cells. **(A)** SCC25 cells with stable STAT3 overexpression or control cells were established and subjected to RT-PCR and Western blot analysis. **(B)** Images of the wound closure of monolayer SCC25 cells with STAT3 overexpression at the time point of 0 and 24 h are presented on the left. Quantitative results are illustrated on the right. **(C)** The effect of STAT3 overexpression on OSCC cells invasion were determined by Transwell assay with Matrigel, and the representative images are on the left. Quantitative results are illustrated on the right. Each assay was carried out in triplicate. Results were shown as means ± SD. ^*^*P* < 0.05.

Supplementary Figure 3 Representative micrographs of negative controls using IgG in OSCC tissues by immunohistochemistry. Magnifications: 100× for the left; 400× for the right.

Supplementary Data Specific primers used for real-time PCR (5′-3′).

## References

[1] MassaSTOsazuwa-PetersNChristopherKMArnoldLDSchootmanMWalkerRJ. Competing causes of death in the head and neck cancer population. Oral Oncol. (2017) 65:8–15. 10.1016/j.oraloncology.2016.12.00628109473

[2] MorrisLGChandramohanRWestLZehirAChakravartyDPfisterDG. The molecular landscape of recurrent and metastatic head and neck cancers: insights from a precision oncology sequencing platform. JAMA Oncol. (2016) 3:244–55. 10.1001/jamaoncol.2016.179027442865PMC5253129

[3] SamanDM. A review of the epidemiology of oral and pharyngeal carcinoma: update. Head Neck Oncol. (2012) 4:1. 10.1186/1758-3284-4-122244087PMC3292826

[4] ChenYJChangJTLiaoCTWangHMYenTCChiuCC. Head and neck cancer in the betel quid chewing area: recent advances in molecular carcinogenesis. Cancer Sci. (2008) 99:1507–14. 10.1111/j.1349-7006.2008.00863.x18754860PMC11159516

[5] HowellGMGrandisJR. Molecular mediators of metastasis in head and neck squamous cell carcinoma. Head Neck. (2005) 27:710–7. 10.1002/hed.2022215952195

[6] CavallaroUChristoforiG. Multitasking in tumor progression: signaling functions of cell adhesion molecules. Ann N Y Acad Sci. (2004) 1014:58–66. 10.1196/annals.1294.00615153420

[7] ThompsonEWNewgreenDFTarinD. Carcinoma invasion and metastasis: a role for epithelial-mesenchymal transition? Cancer Res. (2005) 65:5991–5; discussion 5. 10.1158/0008-5472.CAN-05-061616024595

[8] LarueLBellacosaA. Epithelial-mesenchymal transition in development and cancer: role of phosphatidylinositol 3' kinase/AKT pathways. Oncogene. (2005) 24:7443–54. 10.1038/sj.onc.120909116288291

[9] LeeMYoonJH. Metabolic interplay between glycolysis and mitochondrial oxidation: the reverse Warburg effect and its therapeutic implication. World J Biol Chem. (2015) 6:148–61. 10.4331/wjbc.v6.i3.14826322173PMC4549759

[10] GuillaumondFIovannaJLVasseurS. Pancreatic tumor cell metabolism: focus on glycolysis and its connected metabolic pathways. Arch Biochem Biophys. (2014) 545:69–73. 10.1016/j.abb.2013.12.01924393743

[11] WangYShenYWangSShenQZhouX. The role of STAT3 in leading the crosstalk between human cancers and the immune system. Cancer Lett. (2018) 415:117–28. 10.1016/j.canlet.2017.12.00329222039PMC5748258

[12] ChaiEZShanmugamMKArfusoFDharmarajanAWangCKumarAP. Targeting transcription factor STAT3 for cancer prevention and therapy. Pharmacol Ther. (2016) 162:86–97. 10.1016/j.pharmthera.2015.10.00426478441

[13] YuHLeeHHerrmannABuettnerRJoveR. Revisiting STAT3 signalling in cancer: new and unexpected biological functions. Nat Rev Cancer. (2014) 14:736–46. 10.1038/nrc381825342631

[14] ZhangXYLiMSunKChenXJMengJWuL. Decreased expression of GRIM-19 by DNA hypermethylation promotes aerobic glycolysis and cell proliferation in head and neck squamous cell carcinoma. Oncotarget. (2015) 6:101–15. 10.18632/oncotarget.268425575809PMC4381581

[15] LiMJinRWangWZhangTSangJLiN. STAT3 regulates glycolysis via targeting hexokinase 2 in hepatocellular carcinoma cells. Oncotarget. (2017) 8:24777–84. 10.18632/oncotarget.1580128445971PMC5421887

[16] WangTXZhangZQCongYShiXYLiuYHZhaoFL. Prosapogenin A induces apoptosis in human cancer cells *in vitro* via inhibition of the STAT3 signaling pathway and glycolysis. Oncol Lett. (2013) 6:1323–8. 10.3892/ol.2013.156124179517PMC3813670

[17] GujralTSChanMPeshkinLSorgerPKKirschnerMWMacBeathG. A noncanonical Frizzled2 pathway regulates epithelial-mesenchymal transition and metastasis. Cell. (2014) 159:844–56. 10.1016/j.cell.2014.10.03225417160PMC4243058

[18] LuJTanMCaiQ. The Warburg effect in tumor progression: mitochondrial oxidative metabolism as an anti-metastasis mechanism. Cancer Lett. (2015) 356(2 Pt A):156–64. 10.1016/j.canlet.2014.04.00124732809PMC4195816

[19] MaWFuentesGShiXVermaCRaddaGKHanW. FoxO1 negatively regulates leptin-induced POMC transcription through its direct interaction with STAT3. Biochem J. (2015) 466:291–8. 10.1042/BJ2014110925510553

[20] ChenJHuangQWangF. Inhibition of FoxO1 nuclear exclusion prevents metastasis of glioblastoma. Tumour Biol. (2014) 35:7195–200. 10.1007/s13277-014-1913-124771221

[21] ZhangPTuBWangHCaoZTangMZhangC. Tumor suppressor p53 cooperates with SIRT6 to regulate gluconeogenesis by promoting FoxO1 nuclear exclusion. Proc Natl Acad Sci USA. (2014) 111:10684–9. 10.1073/pnas.141102611125009184PMC4115576

[22] YuHKortylewskiMPardollD. Crosstalk between cancer and immune cells: role of STAT3 in the tumour microenvironment. Nat Rev Immunol. (2007) 7:41–51. 10.1038/nri199517186030

[23] HauraEBTurksonJJoveR. Mechanisms of disease: insights into the emerging role of signal transducers and activators of transcription in cancer. Nat Clin Pract Oncol. (2005) 2:315–24. 10.1038/ncponc019516264989

[24] ChangSMHuWW. Long non-coding RNA MALAT1 promotes oral squamous cell carcinoma development via microRNA-125b/STAT3 axis. J Cell Physiol. (2018) 233:3384–96. 10.1002/jcp.2618528926115

[25] YangJGLuRYeXJZhangJTanYQZhouG. Icaritin reduces oral squamous cell carcinoma progression via the inhibition of STAT3 signaling. Int J Mol Sci. (2017) 18:132. 10.3390/ijms1801013228085115PMC5297765

[26] LiXDingRHanZMaZWangY. Targeting of cell cycle and let-7a/STAT3 pathway by niclosamide inhibits proliferation, migration and invasion in oral squamous cell carcinoma cells. Biomed Pharmacother. (2017) 96:434–42. 10.1016/j.biopha.2017.09.14929031202

[27] WangYGuoWLiZWuYJingCRenY. Role of the EZH2/miR-200 axis in STAT3-mediated OSCC invasion. Int J Oncol. (2018) 52:1149–64. 10.3892/ijo.2018.429329532870PMC5843395

[28] PranadaALMetzSHerrmannAHeinrichPCMuller-NewenG. Real time analysis of STAT3 nucleocytoplasmic shuttling. J Biol Chem. (2004) 279:15114–23. 10.1074/jbc.M31253020014701810

[29] LiuLMcBrideKMReichNC. STAT3 nuclear import is independent of tyrosine phosphorylation and mediated by importin-alpha3. Proc Natl Acad Sci USA. (2005) 102:8150–5. 10.1073/pnas.050164310215919823PMC1149424

[30] GkouverisINikitakisNAvgoustidisDKaranikouMRassidakisGSklavounouA. ERK1/2, JNK and STAT3 activation and correlation with tumor differentiation in oral SCC. Histol Histopathol. (2017) 32:1065–76. 10.14670/hh-11-86828090628

[31] Vander HeidenMGCantleyLCThompsonCB. Understanding the Warburg effect: the metabolic requirements of cell proliferation. Science. (2009) 324:1029–33. 10.1126/science.116080919460998PMC2849637

[32] CairnsRAHarrisISMakTW. Regulation of cancer cell metabolism. Nat Rev Cancer. (2011) 11:85–95. 10.1038/nrc298121258394

[33] HuangHTindallDJ. Dynamic FoxO transcription factors. J Cell Sci. (2007) 120 (Pt 15):2479–87. 10.1242/jcs.00122217646672

[34] JiangGHuangCLiJHuangHJinHZhuJ. Role of STAT3 and FOXO1 in the divergent therapeutic responses of non-metastatic and metastatic bladder cancer cells to miR-145. Mol Cancer Ther. (2017) 16:924–35. 10.1158/1535-7163.MCT-16-063128223425PMC5418086

[35] AghazadehSYazdanparastR. Mycophenolic acid potentiates HER2-overexpressing SKBR3 breast cancer cell line to induce apoptosis: involvement of AKT/FOXO1 and JAK2/STAT3 pathways. Apoptosis. (2016) 21:1302–14. 10.1007/s10495-016-1288-427651367

[36] OhHMYuCRGolestanehNAmadi-ObiALeeYSEseonuA. STAT3 protein promotes T-cell survival and inhibits interleukin-2 production through up-regulation of Class O Forkhead transcription factors. J Biol Chem. (2011) 286:30888–97. 10.1074/jbc.M111.25350021730069PMC3162449

[37] WuJBShaoCLiXLiQHuPShiC. Monoamine oxidase A mediates prostate tumorigenesis and cancer metastasis. J Clin Invest. (2014) 124:2891–908. 10.1172/JCI7098224865426PMC4071401

[38] KimTHJoSWLeeYSKimYJLeeSCKimWJ. Forkhead box O-class 1 and forkhead box G1 as prognostic markers for bladder cancer. J Korean Med Sci. (2009) 24:468–73. 10.3346/jkms.2009.24.3.46819543511PMC2698194

[39] XiongXTaoRDePinhoRADongXC. Deletion of hepatic FoxO1/3/4 genes in mice significantly impacts on glucose metabolism through downregulation of gluconeogenesis and upregulation of glycolysis. PLoS ONE. (2013) 8:e74340. 10.1371/journal.pone.007434024015318PMC3755981

[40] WilhelmKHappelKEelenGSchoorsSOellerichMFLimR. FOXO1 couples metabolic activity and growth state in the vascular endothelium. Nature. (2016) 529:216–20. 10.1038/nature1649826735015PMC5380221

